The article "Migration and Deposition Law of Pollutants in Urban Sewage Confluence Pipe Network from the Perspective of Ecology" was retracted in 2023. Reasons: signs of a paper mill; suspected computer-generated content; unreliable results or conclusions; concerns about the data.

# Migration and Deposition Law of Pollutants in Urban Sewage Confluence Pipe Network from the Perspective of Ecology

**DOI:** 10.1155/2022/1229636

**Published:** 2022-09-19

**Authors:** Shan Hua, Xingwang Pei, Wenlong Li, Hanlie Cheng, Hailian Zhao, David Sturdivant

**Affiliations:** ^1^College of Civil Engineering, Xi'an University of Architecture & Technology, Xi'an Shaanxi 710055, China; ^2^College of Civil Engineering, Xi'an University of Architecture & Technology Huaqing College, Xi'an Shaanxi 710043, China; ^3^Zhongtian Northwest Construction Investment Group Co., Ltd., Xi'an Shaanxi 710065, China; ^4^School of Energy Resource, China University of Geosciences (Beijing), Beijing 434000, China; ^5^School of Soil and Water Conservation, Beijing Forestry University, Beijing 100083, China; ^6^The King's School, BP1560, Bujumbura, Burundi

## Abstract

Aiming at the problem of pollutant migration and deposition in urban sewage confluence pipe, an experimental simulation system of sewage confluence pipe was established. The confluence conditions of three flow patterns (velocity ratio Vaccess/Vtrunk = 0.1/0.2, Vaccess/Vtrunk = 0.1/0.3, and Vaccess/Vtrunk = 0.2/0.3) were simulated. The changes of sediment thickness, carbon pollutants, nitrogen pollutants, and phosphorus pollutants in different confluence areas were analyzed, and the migration and deposition laws of various pollutants in urban sewage confluence pipe network under different flow patterns were revealed. The results show that when the flow velocity of trunk and branch roads changes, the deposition of various pollutants and the carrying capacity of water flow in the pipeline change, resulting in the change of sediment layer thickness and pollutant content. With the increase of trunk velocity, the sediment thickness in the area before and after confluence decreases, while the increase of branch velocity only reduces the sediment thickness in the area at the back of confluence. Under any flow pattern, the sediment thickness in the retention area (G3 and G4) shows an increasing trend, which is the key area of pollution removal. Under the three flow patterns, the content of carbon pollutants reaches the peak at the TCOD and SCOD values of G4 monitoring point. Increasing the trunk velocity can effectively reduce the content of carbon pollutants. The content of nitrogen pollutants in each flow pattern also reaches the maximum at G4 point, which are 213.6 mg/g, 205.2 mg/g, and 212.8 mg/g, respectively. Increasing the trunk velocity can effectively reduce the nitrogen content at points G1-G4, while increasing the flow velocity of the branch road can reduce the nitrogen content at points G5-G7. The distribution of phosphorus pollutants is complex, and the flow pattern needs to be adjusted according to different monitoring points.

The article "Migration and Deposition Law of Pollutants in Urban Sewage Confluence Pipe Network from the Perspective of Ecology" was retracted in 2023. Reasons: signs of a paper mill; suspected computer-generated content; unreliable results or conclusions; concerns about the data.

## 1. Introduction

With the acceleration of industrialization and urbanization, the domestic and industrial water consumption of residents has increased sharply, which has brought great challenges to the operation of urban sewage pipe network. As a result, the deposition of pipe network system is becoming more and more serious, and the capacity of receiving and discharging sewage is obviously decreased [1–4]. Typically, an urban watershed is a stormwater collecting and conveyance network that is in charge of swiftly collecting rainwater from just urban locations in order to minimize severe floods. Following usage, wastewater is gathered in a system of sewers, or occasionally ditches, that connects to a wastewater treatment facility or disposal location. Prior to actually releasing effluent into receiving reservoirs or onto impervious surfaces, sewage treatment facilities eliminate a portion of the pollutants from the effluent. Urban sewage pipe network plays a very important role in the whole sewage treatment and is the first checkpoint of the sewage treatment system [5]. Because the sewage treatment plant is generally far away from the city, the sewage transportation flow time is long, which contains C, N, P, and other pollutants in the pipeline anaerobic environment which will occur a series of physical and chemical series reactions, resulting in changes in the types, concentrations and properties of pollutants, affecting the subsequent sewage treatment process [6–10]. In addition, there are some problems in the sewage pipeline system, such as mixing of rain and sewage, lack of organic matter, sediment blockage, and toxic and harmful gases, which will inevitably cause environmental pollution, especially the pollution of water resources and endanger people's production and life [11–13]. Therefore, this paper studies the migration and deposition law of pollutants in urban sewage confluence pipe network, in order to provide ideas for the rational design of urban sewage pipe network and pipe cleaning.

As a key link of ecological city, urban sewage pipe network has attracted more and more attention of researchers. Kulandaiyelu et al. evaluated the control effect of iron (Fe3+) salt on the content of organic micropollutants (MPs) in pipe network wastewater by using sewage reactor to simulate sewage pipe network, so as to reduce the discharge of phosphorus and sulfide in wastewater treatment plant (WWTP). The merits of using wastewater treatment are good for the environment, provide processed pure water, a strategy to reduce waste, and help you save money, conserve water, and so on [14]. The presence of phosphorus restricts the development of algae as well as aquatic plants in the majority of subsurface waterways. Consequently, the release of P-loads from industrial wastes often leads in a rise in the formation of microalgae and autotrophs, which can sometimes lead in eutrophication as well as worse water management. Bioactive molecules discovered in freshwater resources and treatment facilities for wastewater at levels of less than a few micrograms per liter are known as organic environmental pollutants. The majority of effluents are bioactive, and most are difficult to biodegrade. Gamage was used to remove 18 different kinds of pollutants from sewage pipe network, taking into account the effectiveness and maximum concentration, biological concentration factor, and half-life of the pollutants in the sewage system. Ozonation, reverse osmosis, electrolysis, ion exchange, and adsorption were used to remove the pollutants, and the removal effects of each technology were evaluated [15]. The Newton-Raphson approach, sometimes referred to as Newton's technique, is a rapid way to locate a reliable estimate for a real-valued function's root. It makes advantage of the notion that in a single direction parallel to a constant, linear interpolation can serve as a rough approximation. Pilotti et al. combined the nonbinary tree access algorithm with the Newton-Raphson method to evaluate the distribution of dissolved oxygen in the drainage network by processing drainage network grid diagram [16]. Liu analyzed the concentration changes of pollutants in the urban drainage pipe network at the water inlet, main pipeline, branch pipeline, and water outlet, as well as the distribution of sewage pipeline sediments under different drainage intensities, which provided a scheme for the optimization of urban drainage pipe network system [17]. In order to clarify the relationship between pollutant concentration and flow velocity, Sang et al. established a sewage simulation system and studied the effects of flow velocity of 0.1, 0.3, 0.6, 0.9, and 1.2 m·s^−1^ on the contents of carbon (organic), nitrogen, and phosphorus in the pipeline [18]. Li et al. proposed a multisensor fusion estimation method based on autoregressive moving average model to simulate and monitor the flow velocity of sewage pipe network system, so as to ensure the smooth flow of sewage and provide convenience for dredging work [19]. Giving precise fundamental information is beneficial for feature-level and decision-level fusion. In feature-level fusion, characteristic knowledge from various sensors is first retrieved, and then, the statistics are examined and analyzed. For real-time analysis, this kind of fusion permits the acquisition of encrypted image.

The article "Migration and Deposition Law of Pollutants in Urban Sewage Confluence Pipe Network from the Perspective of Ecology" was retracted in 2023. Reasons: signs of a paper mill; suspected computer-generated content; unreliable results or conclusions; concerns about the data.

In order to clarify the distribution law of pollutants in urban sewage confluence pipe network, an experimental simulation system of sewage confluence pipe is established. The confluence conditions are simulated under three flow patterns of velocity ratio Vaccess/Vtrunk = 0.1/0.2, Vaccess/Vtrunk = 0.1/0.3, and Vaccess/Vtrunk = 0.2/0.3. The changes of sediment layer thickness and carbon pollutants (TCOD and SCOD, potassium dichromate digestion method), nitrogen pollutants (TN, alkaline potassium persulfate UV spectrophotometry), and phosphorus pollutants (TP, molybdenum antimony antispectrophotometry) at G1-G7 monitoring points under each flow pattern are observed. In order to reveal the migration and deposition laws of various pollutants under different flow patterns in urban sewage confluence pipe network, which provides a theoretical basis for urban pipe network design optimization and sewage pipeline dredging.

## 2. Methods and Materials

The actual sewage pipe network is surrounded by the underground of the city. Affected by the area of the experimental site, it is impossible to simulate the actual length of the urban sewage pipe network. Therefore, in this experimental study, a certain length proportion of simulated pipeline is established to simulate the actual sewage pipe network, and the internal circulation flow is used to meet the requirements of the actual hydraulic retention time. The mean amount of time the material is held within the digestion is known as the hydraulic retention time (HRT). The soil nutrient feed-in per period of time and furnace capacity is used to calculate the ecological loading rates (OLR) and how long aqueous and hydrophilic substances typically remain in a burner or container. It is computed by splitting the reactor's capacity (in m^3^) through the speed of initial concentration flow (in m^3^/day). This research is carried out from the following points: (1) design of experimental simulation system for sewage confluence pipeline. The device is shown in Figure 1. (2) Set the experimental conditions. The experiment was divided into three groups: Vaccess/Vtrunk = 0.1/0.2, Vaccess/Vtrunk = 0.1/0.3, and Vaccess/Vtrunk = 0.2/0.3. The first group was operated for 90 days, and the experimental period of adjusting the flow velocity of trunk roads and branches was 30 days. The sewage used in the experiment was sewage at the entrance of Qingdao Younuo wastewater treatment plant. In order to improve the accuracy of the experiment, urban sewage was replaced daily [20–25]. The experimental sewage is pumped to the inlet tank of the system through the submersible sewage pump, the confluence state is simulated by the lift pump, the sewage flow of the branch and trunk is controlled by the regulating valve, and the combined sewage enters the outlet tank to complete the sewage simulation experiment. Ozone, chlorine, UV radiation, and sodium hypochlorite are often used disinfectants. Due to its durability, monochloramine, which is employed to cleanse groundwater, is not utilized to treat wastewater [26–28]. (3) Determine the location of monitoring points. Seven sampling points are set in the experiment, which are located in different confluence areas. In particular, scores of pollutions caused, including unsupervised source information, spirals, waterways, low-pressure regions, and framework finishes, ought to be included in this list of locations because they provide sample population of the circumstances at the resource program's least favorable references or areas [29–31]. The specific location is shown in Figure 2. (4) Sampling. After the end of the experimental operation cycle, close the pipe valve, open the sampling port after the system is stable, the sample is stored at low temperature. (5) Indicator determination. The indicators of carbon pollutants TCOD and SCOD, nitrogen pollutants TN, and phosphorus pollutants TP were determined by potassium dichromate digestion method, alkaline potassium persulfate UV spectrophotometry, and molybdenum antimony antispectrophotometry [32–35]. The solubility COD in the bioreactor is represented by SCOD, whereas the overall COD in the bioreactor is represented by TCOD. When evaluating microorganism responses to atmospheric alterations throughout most of the acclimatization period, COD fluctuations are crucial. Among the most frequently utilized different chemicals in organometallic chemistry are soluble in dilute. It is largely used in labs and in the industry as a potent oxidizing agent in a variety of molecular processes. Anywhere oxidizing is concerned, potassium dichromate is a crucial reagent that is frequently employed. Whenever a blank result is greater than usual, the ammonium hydroxide persulfate digesting UV spectrophotometric technique is typically used to determine the total ammonia in freshwater. The molybdenum blue phosphorus technique combined with a UV-visible spectrometer is used to quantify the quantity of phosphorous. This approach is predicated on the creation of phosphomolybdate combination with the addition of molybdate, accompanied by the degradation of the compound with hydrazine in an environment of dilute sulfuric acid.

The article "Migration and Deposition Law of Pollutants in Urban Sewage Confluence Pipe Network from the Perspective of Ecology" was retracted in 2023. Reasons: signs of a paper mill; suspected computer-generated content; unreliable results or conclusions; concerns about the data.

## 3. Results and Analysis

### 3.1. Sediment Layer Thickness

In order to make the simulation system of urban sewage pipe network more authentic and effective, the reactor needs to run for 3 months (90 d) under the environment of velocity ratio Vaccess/Vtrunk = 0.1/0.2 before the experiment, so that each sampling point (G1-G7) in the pipeline has a certain deposition of particulate pollutants, so as to improve the accuracy of the simulation experiment. During the 90 d-150 d operation of the simulator, the velocity ratio is adjusted from Vaccess/Vtrunk = 0.1/0.2 to Vaccess/Vtrunk = 0.1/0.3, and during 150 d-210 d, the velocity ratio is adjusted from Vaccess/Vtrunk = 0.1/0.3 to Vaccess/Vtrunk = 0.2/0.3. The variation of sediment thickness at each sampling point under different confluence conditions was observed, as shown in Figure 3. At the initial stage of operation of the urban sewage pipe network simulation system, the velocity ratio is Vaccess/Vtrunk = 0.1/0.2, the sewage flow capacity is weak, and the deposition rate of particulate pollutants in sewage under the action of gravity is greater than the migration rate. At 90 days, the sediment thickness of G1-G7 is 60.3 mm, 64.2 mm, 62.3 mm, 58.6 mm, 61.1 mm, 63.0 mm, and 62.9 mm, respectively. Whenever water corrodes the sediment around the foundation or associated structures of bridges, highways, and other man-made constructions, scour develops. Scour is frequently brought on by swift water movement; hence, it frequently happens throughout storms. During the period of 90 d-150 d, the increase of sewage flow velocity on the trunk road strengthens the scouring effect of water on pipeline sediments, and the thickness of sediments in G1-G7 area changes to varying degrees. As G3 and G4 areas are located at the junction of branch roads and trunk roads, the sediment thickness in this area increases slightly by 2-5 mm due to the impact of two streams of water, and the sediment thickness in other areas decreases. G1 and G2 are located at the front of confluence, and the thickness decreases by 10.4 mm and 7.9 mm, respectively, and the sediment thickness at G6 and G7 decreases slightly by about 6 mm. The change is most significant at G5, and its thickness is reduced by 14.2 mm. During 150 d-210 d, the velocity ratio is adjusted from Vaccess/Vtrunk = 0.1/0.3 to Vaccess/Vtrunk = 0.2/0.3. Due to the increase of sewage flow rate in the branch, the carrying capacity of water body to pollutant particles is enhanced, but the pipe diameter of the branch is small and the influence range is limited. Therefore, the sediment thickness at the front of confluence (G1 and G2) and confluence area (G3 and G4) increases, while the sediment thickness at G5, G6, and G7 decreases slightly by 6.1 mm, 4.5 mm, and 3.8 mm, respectively.

The article "Migration and Deposition Law of Pollutants in Urban Sewage Confluence Pipe Network from the Perspective of Ecology" was retracted in 2023. Reasons: signs of a paper mill; suspected computer-generated content; unreliable results or conclusions; concerns about the data.

Therefore, when the flow velocity of trunk and branch roads changes, the deposition of particulate pollutants in the pipeline and the carrying capacity of water flow change accordingly, resulting in the increase or decrease of sediment thickness. According to the change of sediment thickness and the location of branch and trunk roads, the monitoring points G1-G7 are divided. G1 and G2 are the front end of the confluence, G3 and G4 are the retention area, G5 is the separation area, and G6 and G7 are the back end of the confluence. When the flow velocity of sewage in the trunk road increases, the sediment thickness in the area before and after confluence decreases. When dirt is removed from the area surrounding a pile foundation for a highway or an offshore structure, the organization's ability is decreased in both the lateral and vertical directions. From the river's greatest water level, the average scour depth is calculated. To determine the mean velocity of the fluid of the channel, increase the surface water flow rate (in m/s) by 0.85 (a compensation element) and divide the outcome by the length from point A to point B (10 m in this instance). When the flow velocity of sewage in the branch road increases, the sediment thickness increases in the front area of confluence and decreases in the back area of confluence, but the decreasing trend of this thickness is not obvious compared with increasing the flow velocity of trunk road. Under either flow pattern, the thickness of the sediment in the fluid confluence retention area shows an increasing trend, which is the focus area of the cleaning work. The flawless interior surfaces of sewage begin to be damaged by solid matter particles when the flow rate surpasses a specific threshold, or in simpler phrases, a scouring operation occurs.

### 3.2. Carbon Pollutant Content

The content of carbon organics is the key to the stable operation of the sewage treatment system. The mass lost during the burning of a material is used to calculate the number of particulate hydrocarbons. This may be accomplished in liquid solution by determining the total matter of a filtration that had a given volume of water run across it both before and after the filtration was heated to 550°C for ignition. Therefore, taking TCOD and SCOD as measurement indicators, the contents of carbon organics in the pipeline sedimentary layer in each confluence area under different flow patterns are characterized [36–38].  Table 1 is the variation of TCOD and SCOD in the sedimentary layer under three flow conditions: Vaccess/Vtrunk = 0.1/0.2, Vaccess/Vtrunk = 0.1/0.3, and Vaccess/Vtrunk = 0.2/0.3. Along the flow direction of sewage, TCOD and SCOD showed the same change trend. The contents of TCOD and SCOD in G1-G2 decreased slightly and then increased gradually, reaching the peak at G4 monitoring point. After a significant decrease at G5 in the separation area, the content of carbon pollutants stabilized at the back end of the confluence [39–41]. Taking the velocity ratio Vaccess/Vtrunk = 0.1/0.2 as an example, the contents of average total organic matter TCOD and average dissolved organic matter SCOD in different confluence areas are analyzed. The values of TCOD and SCOD at G1 are 11.1 × 103 mg/g and 250.7 mg/g, respectively. When flowing to G2 monitoring point, the content of both decreased slightly, but the change value was small [42]. When the sewage further flows to point G4 in the retention area, the organic content in each depth of the sedimentary layer reaches the maximum, which is 12.2 × 103 mg/g and 323.8 mg/g, respectively, increased by 10.3% and 29.2% compared with G1 point. After that, the content of organic matter decreased sharply at G5 point in the separation area, decreased by 26.1% and 45.2% to 9.0 × 103 mg/g and 177.6 mg/g, respectively. At the back end of the confluence, the content of carbon pollutants tends to be stable, and the carbon index values are 7.3 × 103 mg/g (RTCOD) and 142.0 mg/g (RTCOD), respectively, decreased by 33.8% and 43.4% compared with G1 point.

The article "Migration and Deposition Law of Pollutants in Urban Sewage Confluence Pipe Network from the Perspective of Ecology" was retracted in 2023. Reasons: signs of a paper mill; suspected computer-generated content; unreliable results or conclusions; concerns about the data.

Increase the flow velocity of trunk sewage pipe; that is, when the velocity ratio is adjusted from Vaccess/Vtrunk = 0.1/0.2 to Vaccess/Vtrunk = 0.1/0.3, the TCOD content shows a downward trend in each confluence area, and the largest decline in the separation area G5 is 2.56 × 10^3^ mg/g, followed by G6 (1.72 × 10^3^ mg/g), G2 (1.19 × 10^3^ mg/g), and G7 (1.13 × 10^3^ mg/g); the decline in the monitoring point is less than 1 × 10^3^ mg/g. Except for the increase of G3 and G4 in the retention area, the SCOD value also showed a downward trend at the monitoring points. When the velocity ratio is adjusted from Vaccess/Vtrunk = 0.1/0.3 to Vaccess/Vtrunk = 0.2/0.3 to increase the branch flow velocity, the RTCOD and RSCOD in the front end of confluence and retention area increase, but the overall increase is not obvious, and the carbon pollutant content in separation area decreases, while the RTCOD values of G6 and G7 in the back end of confluence decrease by 0.26 × 10^3^ mg/g and 0.69 × 10^3^ mg/g, respectively, while SCOD increase by 11.12 mg/g and 7.71 mg/g.

### 3.3. Nitrogen Pollutants

Figure 4 shows the changes of nitrogen content in sedimentary layers in each confluence area under three flow patterns: velocity ratio Vaccess/Vtrunk = 0.1/0.2, Vaccess/Vtrunk = 0.1/0.3, and Vaccess/Vtrunk = 0.2/0.3. The content of nitrogen pollutants showed an upward trend in the front of the confluence and the retention area under the three flow patterns. Among them, the G2-G3 interval increased greatly from 130.4 mg/g to 189.4 mg/g under the condition of velocity ratio Vaccess/Vtrunk = 0.1/0.3. Under the three flow patterns, the nitrogen content reached the maximum at G4 point, which were 213.6 mg/g, 205.2 mg/g, and 212.8 mg/g, respectively. There was a significant decrease in the separation area, with the decrease rates of 61.3%, 55.7%, and 60.7%, respectively. When the sewage passes through the back end area of the confluence, the TN value rises slightly and finally stabilizes at about 92 mg/g, 100 mg/g, and 93 mg/g, which are decreased by 40.8%, 22.1%, and 39.4%, respectively, compared with the G1 point. With the increase of the flow velocity of the trunk pipeline, the velocity ratio was adjusted from Vaccess/Vtrunk = 0.1/0.2 to Vaccess/Vtrunk = 0.1/0.3. The nitrogen content in the front end of the confluence decreased significantly, and the G1 and G2 points decreased by 26.1 mg/g and 45.6 mg/g, respectively. The TN in the retention area decreased slightly, and the nitrogen pollutant content in the separation area and the back end of the confluence increased. The overall change was small, and the increase was less than 10 mg/g. After the branch flow velocity was increased, the velocity ratio was Vaccess/Vtrunk = 0.2/0.3, and the TN value of G1-G4 showed an upward trend. In particular, the increase in the front end of the confluence was particularly obvious, and the nitrogen content at the monitoring point decreased.

The article "Migration and Deposition Law of Pollutants in Urban Sewage Confluence Pipe Network from the Perspective of Ecology" was retracted in 2023. Reasons: signs of a paper mill; suspected computer-generated content; unreliable results or conclusions; concerns about the data.

### 3.4. Phosphorus Pollutants

Figure 5 shows the changes of phosphorous content in sedimentary layers in each confluence area under three flow patterns: velocity ratio Vaccess/Vtrunk = 0.1/0.2, Vaccess/Vtrunk = 0.1/0.3, and Vaccess/Vtrunk = 0.2/0.3. Compared with the distribution of nitrogen pollutants, the distribution of phosphorus pollutants is more complex. Under the condition of velocity ratio Vaccess/Vtrunk = 0.1/0.2, along the direction of sewage flow, the TP value increased slightly at the front end of the confluence and then decreased to the retention area. After jumping to the maximum value of 113.4 mg/g at G5 point, the phosphorus content decreased significantly to a stable state, and the TP values of G6 and G7 were about 44 mg/g. The distribution of phosphorus pollutants under the condition of velocity ratio Vaccess/Vtrunk = 0.1/0.3 is the same as that of Vaccess/Vtrunk = 0.1/0.2, but the spatial fluctuation is small. Under the condition of velocity ratio Vaccess/Vtrunk = 0.2/0.3, the phosphorus content in the G1-G3 interval showed a downward trend, which increased slightly at G4 and then decreased again, and finally stabilized at about 56 mg/g. After increasing the flow velocity of sewage in trunk roads, the phosphorus pollutant content at monitoring points decreased significantly except for a small increase in TP value at the back end of confluence. After increasing the branch flow velocity, the TP value of G1 and G4 points increased significantly.

The article "Migration and Deposition Law of Pollutants in Urban Sewage Confluence Pipe Network from the Perspective of Ecology" was retracted in 2023. Reasons: signs of a paper mill; suspected computer-generated content; unreliable results or conclusions; concerns about the data.

## 4. Conclusion

1. When the flow velocity of sewage in the trunk road increased, the sediment thickness in the area before and after the confluence decreased. When the flow velocity of sewage in the branch road increased, the sediment thickness increased in the front end of the confluence area and decreased in the back end of the confluence area. Regardless of the flow pattern, the thickness of the sediment in the fluid confluence retention areas (G3 and G4) showed an increasing trend, which was the key area of pollution removal
2. The TCOD and SCOD values of carbon pollutants reached the peak at G4 monitoring point, and the content of carbon pollutants could be effectively reduced by increasing the trunk velocity. The maximum decrease was 2.56 × 10^3^ mg/g at G5, followed by G6 (1.72 × 10^3^ mg/g), G2 (1.19 × 10^3^ mg/g), and G7 (1.13 × 10^3^ mg/g)
3. Under the three flow patterns, the nitrogen content reached the maximum at G4, which were 213.6 mg/g, 205.2 mg/g, and 212.8 mg/g, respectively. Increasing the trunk flow velocity can effectively reduce the nitrogen content at G1-G4, while increasing the branch flow velocity can reduce the nitrogen content at G5-G7
4. The distribution of phosphorus pollutants is relatively complex. After increasing the flow velocity of the trunk road, the content of phosphorus pollutants in other monitoring points decreased significantly, except that the TP value in the back end of confluence increased slightly. After increasing the flow velocity of the branch road, the TP value of G1 and G4 increased significantly

## Figures and Tables

**Figure 1:** Schematic diagram of sewage confluence pipeline simulation system.

**Figure 2:** Distribution diagram of sampling points in confluence area.

**Figure 3:** Variation of sediment thickness in each confluence area under different sink states.

**Figure 4:** Variation of nitrogen content in sedimentary layers of each confluence area under different flow patterns.

**Figure 5:** Variation of phosphorus content in sedimentary layer of each confluence area under different flow patterns.

**Table 1:** RTCOD and RSCOD values of sediment in each confluence area under different flow patterns.

Confluence area		G1	G2	G3	G4	G5	G6	G7
Vaccess/Vtrunk = 0.1/0.2	TCOD (10^3^mg/g)	11.0	10.4	11.0	12.2	9.0	7.5	7.3
	SCOD (mg/g)	250.7	231.1	282.6	323.8	177.6	141.5	142.0
Vaccess/Vtrunk = 0.1/0.3	TCOD (10^3^mg/g)	10.3	9.2	10.9	11.9	6.4	5.8	6.2
	SCOD (mg/g)	217.5	183.0	291.9	332.8	136.8	101.2	100.3
Vaccess/Vtrunk = 0.2/0.3	TCOD (10^3^mg/g)	11.1	10.3	11.7	12.7	5.9	5.5	5.5
	SCOD (mg/g)	231.3	207.7	334.9	366.7	123.6	112.3	108.0
Increase trunk flow rate	TCOD difference	-0.74	-1.19	-0.15	-0.30	-2.56	-1.72	-1.13
	SCOD difference	-33.18	-48.14	9.29	9.02	-40.80	-40.35	-42.00
Increase branch flow rate	TCOD difference	0.79	1.08	0.80	0.85	-0.54	-0.26	-0.69
	SCOD difference	13.77	24.70	42.97	33.86	-13.21	11.12	7.71

The article "Migration and Deposition Law of Pollutants in Urban Sewage Confluence Pipe Network from the Perspective of Ecology" was retracted in 2023. Reasons: signs of a paper mill; suspected computer-generated content; unreliable results or conclusions; concerns about the data.

## Data Availability

The figures and tables used to support the findings of this study are included in the article.
